# Prevalence and Complications of Glycogen Storage Disease in South Korea: A Nationwide Population-Based Study, 2007-2018

**DOI:** 10.1155/2022/2304494

**Published:** 2022-07-01

**Authors:** Eun Jung Lee, Ha Eun Chang, Sung Hwa Kim, Yong Whi Jeong, Hong Koh, Yunkoo Kang

**Affiliations:** ^1^Department of Pediatrics, Yonsei University Wonju College of Medicine, Wonju, Republic of Korea; ^2^Yonsei University Wonju College of Medicine, Wonju, Republic of Korea; ^3^Department of Biostatistics, Yonsei University Wonju College of Medicine, Wonju, Republic of Korea; ^4^Department of Pediatrics, Yonsei University College of Medicine, Seoul, Republic of Korea

## Abstract

Glycogen storage disease (GSD) is a rare disease that can cause life-threatening problems owing to metabolic errors in storing or using glycogen. The disease course of GSD remains unknown, despite medical technology advances. We determined the prevalence and complications of GSD using data from the National Health Insurance Service database. Data were collected and analyzed for the entire South Korean population with GSD during 2007–2018. GSD was defined as a combination of disease code E74.0 and rare incurable disease insurance code V117, a unique disease code combination for GSD in South Korea. Overall, 23,055 patients had the E74 disease code; 404 had an additional V117 insurance code. Most GSD patients were aged <10 years. Many complications were identified, the most common being hepatomegaly, hyperuricemia, and elevated liver enzyme levels. The most prescribed drug was *α*-glucosidase, followed by allopurinol. Seventy-two percent of patients were treated in pediatrics. Twenty-five patients underwent liver transplantation, and 14 died after GSD diagnosis. In South Korea, more patients than expected had GSD diagnosis and were managed accordingly. GSD causes many complications and hospitalizations, resulting in high medical expenses. Serious complications can result in liver transplantation and, eventually, death in some cases. Although the patients' condition was identified only by the disease code, this is the first study to present the current situation of GSD patients in South Korea. Because GSD patients can have dangerous medical conditions, they should be managed consistently while minimizing various complications that may occur with optimal metabolic control.

## 1. Introduction

Glycogen storage disease (GSD) is a rare disease that can cause life-threatening problems owing to metabolic errors in storing or using glycogen in the liver or muscle [1]. Furthermore, GSD was first reported by Von Gierke in 1929 in children whose liver and kidneys contained excessive amounts of glycogen; since then, many types of GSD have been described [2]. In Korea, based on single center data, it was confirmed that most of the GSD Ia patients had c.648G > T G6PC mutation in 86.2%, which was similar to 86.4% in Japanese patient cohort and different from the 36% known in Chinese patients [3]. In addition, SLC37A4 mutation was confirmed in GSD Ib patients, PHKA2 mutation spectrum in type IX patients, and AGL mutation spectrum in type III patients to understand the characteristics of Korean glycogen storage disease patients [4–6]. However, prevalence and types of GSD in South Koreans has not yet been described through a large-scale investigation. Additionally, although the administration of corn starch has recently been established as a standard treatment method, it is not possible to predict which complications would arise in the future because there are no large-scale data in South Korea [7, 8].

Therefore, in this study, we investigated the prevalence of GSD in South Korea and possible complications and problems in GSD for more efficient treatment.

## 2. Methods

### 2.1. Study Design

The National Health Insurance system provides all medical information of the population in South Korea. Furthermore, the Health Insurance and Review Assessment Service (HIRA) has every medical database available for researchers. This retrospective, population-based cohort study was conducted using HIRA research data.

South Korea defines GSD as a rare disease and provides financial support by registering the rare incurable disease insurance code V117, a unique disease code for patients with GSD in South Korea. When registering V117, laboratory tests, genetic tests, and doctor's judgment are required. We tried to define patients with GSD as having a combination of both disease codes E74.0 and V117.

We obtained medical records of patients with GSD during 2007–2018. Among patients with GSD, we defined patients as having complications according to the International Classification of Diseases (ICD) codes other than E74.0.

The Institutional Review Board of Wonju Severance Christian Hospital approved this study (IRB No. CR319323).

### 2.2. Statistical Analyses

Data were expressed according to variable characteristics. Categorical data are reported as numbers with percentages and were compared using Pearson's chi-square test or Fisher's exact test. Continuous data are reported as means ± standard deviations and were compared using independent *t*-test or Mann-Whitney *U* test.

Chi-square tests were used to detect any differences in the distribution of numbers and costs according to age, sex, and disease codes. The annual number of each procedure and its crude incidence, that is, the GSD patients/year-specific population, was calculated. Annual population data of South Koreans were obtained from the Korean Statistical Information Service. Data analysis was performed using SAS software (version 9.4). A *p* value of < 0.05 was considered to indicate statistical significance for all analyses.

## 3. Results

### 3.1. Baseline Characteristics (2020-10-06 Section)

Overall, 23,055 patients had the ICD code E74 during 2007–2018. Among them, 741 (3.21%) had only the ICD code E74.0, and 404 (1.7%) had both E74.0 and V117 codes (Figure 1).

From 2007 to 2018, 404 patients with GSD were classified by age (Table 1). The mean patient age was 16.29 years, and 254 males and 150 females were included.

### 3.2. Prevalence of GSD

A graph of the age-adjusted rate of newly diagnosed GSD cases since 2007 is shown in Figure 2(a). The crude rate of GSD diagnosis by age since 2007 is shown in Figure 2(b). The initial rate was high because the registration of the rare incurable disease insurance code V117 started in 2007. The age-adjusted rate of newly diagnosed cases was between 0.03 and 0.08, and most of the patients were diagnosed under the age of 9 years. Years 2007 and 2008 are the washout periods as it was affected by previously diagnosed GSD which may confound the incidence of GSD in Korea. From 2009 to 2018, the incidence of GSD in Korea is 0.05 cases/100,000 persons.

### 3.3. Managing GSD Patients

After diagnosis, 71% of the patients were managed by a pediatrician in 2018 (Table 2). Patients with GSD tend to be managed by pediatricians, even when they are older.

In 2018, 363 patients with GSD visited hospital in Korea. A total of 261 admissions and 2,266 outpatient clinic visits were conducted. In 2018, the average medical cost per patient was 30,601,989 won. There was a difference, from a minimum of 16,890 won to a maximum of 752,667,350 won. From 2007 to 2018, the average total hospital cost of 404 patients with GSD was 169,730,862 won, which varied from a minimum of 256,740 won to a maximum of 3,525,930,160 won.

### 3.4. Complications of Patients with GSD

Among the complications, the hepatomegaly code was the most frequently included code in the data. Furthermore, hyperuricemia and elevation of liver enzymes, followed by growth failure, hypoglycemia, cardiac hypertrophy, hypertriglyceridemia, and hematuria, were the most common complications of GSD (Table 3).

### 3.5. Medication of Patients with GSD

Various medications were prescribed to patients with GSD in 2018. The most prescribed medication for GSD was alpha-glucosidase, which is used for GSD II. Filgrastim was the next most prescribed treatment, and it was is thought to be for patients with GSD Ib. Allopurinol was widely administered to patients with GSD.

### 3.6. Liver Transplantation

Twenty-five patients (14 males, 11 females) received liver transplantation after the diagnosis of GSD despite receiving various treatments. The average age at liver transplantation was 19.24 years (male, 20.07; female, 18.18 years). Since 2007, 14 patients have died of GSD complications. The average age was 25.43 years (male 27.5, female 23.29 years). Among the 14 patients, patients died at approximately 1,048 days after being diagnosed with GSD (minimum, 59 days; maximum, 3785 days).

## 4. Discussion

This study described the current status of patients with GSD disease codes in South Korea, including age at diagnosis, number of hospitalizations and outpatient visits, medical expenses, complications, and mortality.

Although it was not possible to distinguish the exact type of GSD patients, a total of 404 people were diagnosed with GSD in South Korea from 2007 to 2018, of whom 224 (56%) were diagnosed before the age of 9 years with the development of diagnostic technology and efforts of medical staff. However, most patients with GSD receive outpatient and inpatient treatment and spent an average of 30 million won a year, which increases medical expenses and leads to many complications.

Rake et al. described the complications of 231 GSD Ia and 57 GSD Ib patients at 16 centers in 12 European countries in 1996 [9, 10]. According to them, complications due to hyperuricemia were observed in 14% of patients, hepatomegaly in 89% of patients, and splenomegaly in 11% and 49% of GSD1a and GSD 1b patients, respectively. Liver adenoma was also identified in 16% of the patients and was detected at an average age of 15 years. Furthermore, multiple liver adenomas were identified in 64% of patients. Moreover, 50% of cases had progression (increase in size and increase in number), 6 were accompanied by serious complications, 3 involved liver resection, and 2 involved liver transplantation due to complications. These results are similar to the current status of South Korean patients with GSD confirmed in this study.

However, recently, treatment using raw corn starch and maintenance of optimal metabolic control can reduce complications [11]. Complications such as focal hepatic lesion, mild renal dysfunction, and anemia occurred less frequently, and at an earlier stage, raw corn starch treatment was started [1, 12, 13]. Dambska et al. described that the complications of GSD patients can be decreased by optimizing the corn starch dose [14]. Dahlberg et al. reported a sample of corn starch doses of GSD patients and how glucose stabilizes with managing the dose of corn starch [15]. Furthermore, controversies are ongoing about dietary management, although there is consensus regarding managing right for GSD patients [16]. Recently, research on GSD has increased, which confirmed that by consuming an appropriate amount of starch, it is possible to control blood sugar and uric acid levels and to improve various secondary metabolic abnormalities [17].

Therefore, in cases of clinical suspicion, it is necessary to actively conduct related tests; the role of the pediatrician is very important, considering that GSD is diagnosed in individuals belonging to a relatively young age group. Reducing overall complications, medical costs, and mortality through early diagnosis and treatment will be of great help from a social and economic perspective.

Although GSD is a chronic disease that requires lifelong management, not many large-scale analyses have been conducted, and relatively little attention has been paid to it.

As already mentioned in studies conducted in other countries, complications such as hepatomegaly, hyperuricemia, elevated liver enzyme levels, growth failure, hypoglycemia, cardiac hypertrophy, and hyperlipidemia are highly prevalent in South Korean patients with GSD. In addition, it has been confirmed that if proper treatment is not received in time, then hepatic adenomas appear around the age of 10-30 years that become malignant tumors; this may increase the requirement for liver transplantation and may even lead to death.

As described above, GSD is a disease that causes complications accompanied by various metabolic abnormalities, increases the frequency of hospitalization, increases medical expenses, and reduces the quality of life of patients and their families, eventually leading to death.

## 5. Limitation

A limitation of the study is that it confirmed only the disease code without seeing the patient directly. Additionally, there is a high possibility that the frequency of complications may not be accurate because there are many cases in which not all diagnosis names are included when prescribing inpatients and outpatient treatment. The author tried to classify the GSD type but failed in this study. Many attempts were made to classify the GSD type by complication diagnosis code that can be included by each type or a special drug used for each type, but the GSD type could not be distinguished because the diagnosis code was not written properly when treating GSD, and there were cases where proper treatment was not received. This is considered a major limitation in this study. Doctors' efforts should be made to fill in a specific type of patients with glycogen storage disease, complication code rather than just fill in with glycogen storage disease.

In addition, since the registration of rare diseases started in 2007, several patients with GSD were registered between 2007 and 2009, and it may have biased the results. Because the number of previously diagnosed patients has been sufficiently registered, the prevalence rate is expected to be accurate from approximately 2010 onward. Despite these limitations, this is the first study to use big data to confirm the current status of patients with GSD in South Korea.

## 6. Conclusion

In South Korea, more patients than expected are diagnosed with GSD and managed. GSD is associated with many complications and causes frequent hospitalizations, resulting in high medical expenses. Serious complications can result in liver transplantation and even death in some cases. Although there is a limitation that the patient's condition was identified only by the disease code included in the treatment, this is the first study to present the current situation of patients with GSD in South Korea. Because patients with GSD can have dangerous medical conditions, patients with GSD should be managed consistently while minimizing various complications that may occur with optimal metabolic control.

## Figures and Tables

**Figure 1:** Subproportion of patients with the E74 ICD code. ICD: International Classification of Diseases.

**Figure 2:** (a) Age-adjusted rate of newly diagnosed GSD cases by year. GSD: glycogen storage disease. (b) Crude rate of newly diagnosed GSD cases by age. GSD: glycogen storage disease.

**Table 1:** Basic characteristics of GSD patients.

	Total	Male (*n* = 254)	Female (*n* = 150)	*p* value
Mean age (years)	12.89 ± 15.29	11.15 ± 12.76	15.84 ± 18.49	0.0065
Age group (years)				
0–9	226 (0.55)	152 (0.59)	74 (0.49)	
10–19	83 (0.20)	55 (0.21)	28 (0.18)	
20–29	50 (0.12)	28 (0.11)	22 (0.14)	
30–39	19 (0.04)	9 (0.03)	10 (0.06)	
40–49	8 (0.02)	4 (0.02)	4 (0.02)	
50–59	9 (0.02)	3 (0.01)	6 (0.04)	
60–69	3 (0.01)	2 (0.01)	1 (0.01)	
70-79	3 (0.01)	0 (0.0)	3 (0.02)	
80+	3 (0.01)	1 (0.01)	2 (0.01)	

GSD: glycogen storage disease.

**Table 2:** 

Department	Cases (*n*)	Proportion (%)
Pediatrics	287	71.04
Internal medicine	35	8.66
Neurology	29	7.18
General practice	22	5.45
Rehabilitation	16	3.96
General surgery	2	0.5

**Table 3:** Complications of GSD patients.

Complication	Cases (*n*)	Cases/total patient Proportion (%)
Hepatomegaly	51	12.62
Hyperuricemia	36	8.91
Elevated liver enzyme	34	8.42
Growth failure	21	5.20
Hypoglycemia	19	4.70
Cardiomegaly	18	4.46
Hypertriglyceridemia	13	3.22
Hematuria	12	2.97

GSD: glycogen storage disease.

## Data Availability

Access to data is restricted.

## References

[1] Kishnani P. S., Austin S. L., Abdenur J. E. (2014). Diagnosis and management of glycogen storage disease type I: a practice guideline of the American College of Medical Genetics and Genomics. *Genetics in Medicine*.

[2] Von Gierke E. (1929). Hepato-nephro-megalia glycogenica (Glykogenspeicher-krankheit der Leber und Nieren). *Beitrage Zur Pathologischen Anatomie*.

[3] Kim Y. M., Choi J. H., Lee B. H., Kim G. H., Kim K. M., Yoo H. W. (2020). Predominance of the c.648G > T G6PC gene mutation and late complications in Korean patients with glycogen storage disease type Ia. *Orphanet Journal of Rare Diseases*.

[4] Choi R., Park H. D., Ko J. M. (2017). Novel SLC37A4 mutations in Korean patients with glycogen storage disease Ib. *Annals of Laboratory Medicine*.

[5] Choi R., Park H. D., Kang B. (2016). PHKA2 mutation spectrum in Korean patients with glycogen storage disease type IX: prevalence of deletion mutations. *BMC Medical Genetics*.

[6] Ko J. S., Moon J. S., Seo J. K., Yang H. R., Chang J. Y., Park S. S. (2014). A mutation analysis of the AGL gene in Korean patients with glycogen storage disease type III. *Journal of Human Genetics*.

[7] Correia C. E., Bhattacharya K., Lee P. J. (2008). Use of modified cornstarch therapy to extend fasting in glycogen storage disease types Ia and Ib. *The American Journal of Clinical Nutrition*.

[8] Chen Y. T., Bazzarre C. H., Lee M. M., Sidbury J. B., Coleman R. A. (1993). Type I glycogen storage disease: nine years of management with cornstarch. *European Journal of Pediatrics*.

[9] Visser G., Rake J. P., Fernandes J. (2000). Neutropenia, neutrophil dysfunction, and inflammatory bowel disease in glycogen storage disease type Ib: results of the European study on glycogen storage disease type I. *The Journal of Pediatrics*.

[10] Rake J. P., Visser G., Labrune P., Leonard J. V., Ullrich K., Smit G. P. A. (2002). Glycogen storage disease type I: diagnosis, management, clinical course and outcome. Results of the European study on glycogen storage disease type I (ESGSD I). *European Journal of Pediatrics*.

[11] Weinstein D. A., Wolfsdorf J. I. (2002). Effect of continuous glucose therapy with uncooked cornstarch on the long-term clinical course of type 1a glycogen storage disease. *European Journal of Pediatrics*.

[12] Smit G. P. (1993). The long-term outcome of patients with glycogen storage disease type Ia. *European Journal of Pediatrics*.

[13] Talente G. M., Coleman R. A., Alter C. (1994). Glycogen storage disease in adults. *Annals of Internal Medicine*.

[14] Dambska M., Labrador E. B., Kuo C. L., Weinstein D. A. (2017). Prevention of complications in glycogen storage disease type Ia with optimization of metabolic control. *Pediatric Diabetes*.

[15] Dahlberg K. R., Ferrecchia I. A., Dambska-Williams M. (2020). Cornstarch requirements of the adult glycogen storage disease Ia population: a retrospective review. *Journal of Inherited Metabolic Disease*.

[16] Ross K. M., Ferrecchia I. A., Dahlberg K. R., Dambska M., Ryan P. T., Weinstein D. A. (2020). Dietary management of the glycogen storage diseases: evolution of treatment and ongoing controversies. *Advances in Nutrition*.

[17] Ozen H. (2007). Glycogen storage diseases: new perspectives. *World Journal of Gastroenterology*.

